The article "β3-integrin is required for differentiation in OC-2 cells derived from mammalian embryonic inner ear" was published in 2012. Journal: BMC Cell Biol.

# β3-integrin is required for differentiation in OC-2 cells derived from mammalian embryonic inner ear

**DOI:** 10.1186/1471-2121-13-5

**Published:** 2012-03-17

**Authors:** Ivan Brunetta, Stefano O Casalotti, Ian R Hart, Andrew Forge, Louise E Reynolds

**Affiliations:** 1 Centre for Auditory Research, UCL Ear Institute, University College London, London WC1X 8EE, UK; 2 School of Health, Sport and Bioscience, University of East London, London E15 4LZ, UK; 3 Centre for Tumour Biology, Barts Cancer Institute, Queen Mary University of London, Charterhouse Square, London EC1M 6BQ, UK

## Abstract

**Background:**

The mammalian inner ear contains the organ of Corti which is responsible for the conversion of sound into neuronal signals. This specialised epithelial tissue is the product of a complex developmental process where a common precursor cell type differentiates into the sound transducing hair cells and the non-innervated supporting cells. We hypothesised that integrin proteins, which are involved in cell attachment to extracellular matrix proteins and cellular signalling, play a role in the differentiation process of the precursor inner ear epithelial cells. To test our hypothesis we have utilised a cell line (OC-2) derived from E13 embryonic immortomouse inner ears. In vitro, by switching the incubation temperature from 33°C to 39°C, the OC-2 cells can be induced to differentiate and express hair cells markers, such as Myosin VIIa. The OC-2 cells are thus a useful model system for testing mechanism of hair cells differentiation.

**Results:**

We have identified 4 integrin subunits which are expressed in OC-2 cells: α6, αv, β1 and β3. Among these, the relative level of expression of the αv, β1 and β3 subunits increased in a time dependent manner when the cells were exposed to the differentiating temperature of 39°C, most notably so for β3 which was not detectable at 33°C. Treatment of fully differentiated OC-2 cells with siRNA against the four integrin subunits reduced the expression of not only the respective integrin proteins but also of the hair cell marker Myosin VIIa. Conversely over-expression of β3 was sufficient to induce the expression of Myosin VIIa at 33°C.

**Conclusions:**

Our data demonstrate that modulation of integrin expression is associated with the differentiation process of the OC-2 cells. This suggests that the maturation of the organ of Corti, from where OC-2 cells are derived, may also depend on changes of gene expression associated with integrin expression.

## Background

Sound travels as waves of compressed air into the outer ear; it is amplified by the movement of ossicles in the middle ear; and finally is converted into a neuronal signal in the inner ear. In the organ of Corti, sound stimulation of the sensory "hair" cells leads to release of glutamate to initiate neuronal signals which are carried to and processed in the brain. The organ of Corti is a specialised epithelial tissue containing three rows of outer hair cells, one row of inner hair cells and a variety of supporting cells. Each hair cell is surrounded by and separated from its neighbours by intervening supporting cells. The bodies of the supporting cells also intervene between the base of the hair cells and the basilar membrane, the extracellular matrix that underlies the organ of Corti, such that supporting cells, but not hair cells are attached to the basilar membrane. The base of each hair cell is in contact with a nerve terminal where the mechanical sound signal is converted into an electrical nerve signal.

The article "β3-integrin is required for differentiation in OC-2 cells derived from mammalian embryonic inner ear" was published in 2012. Journal: BMC Cell Biol.

The cellular composition and architecture of the organ of Corti is critical to its function [1]. It has been demonstrated that both hair cells and supporting cells are derived from a common precursor [2]. However, the mechanisms of maturation of the organ of Corti are largely unknown [3]. Identification of the factors involved in the differentiation and maturation of the organ of Corti is of interest not only to understand the possible cause of congenital hearing defects but also to understand why the mammalian organ of Corti is unable to regenerate hair when these are killed as a consequence of the effects of damaging agents such as noise or ototoxins or with ageing [4].

During maturation of the organ of Corti, the division of precursor cells into supporting cells and a hair cells is characterised by the detachment of the precursor cells from basilar membrane during the mitotic phase and the formation of the supporting cell that re-attaches to the basilar membrane while the hair cell does not [5,6]. In epithelial tissues, the attachment and detachment of cells to and from the basement membrane is known to be mediated by integrin proteins binding to extracellular matrix protein [7]. Integrins are a family of transmembrane proteins that form heterodimeric surface receptors composed of an α and β subunit [8]. The integrin receptor heterodimers have specific affinities for extracellular proteins commonly found in the basement membrane and, upon binding, they are capable of sending signals which can determine developmental processes in the cells [9,10]. There is evidence that integrins are expressed in the inner ear [11] and that they play an important functional role as demonstrated by the effect of mutations [12]. However, their role in the differentiation and maintenance of the organ of Corti requires further investigation. In this study we have chosen to use a cell line (OC-2) derived from embryonic day 13 (E13) immortomouse inner ear [13]. This cell line has previously been demonstrated to have certain characteristics of developing inner ear epithelial cells. OC-2 cells can be maintained in a proliferative state at 33°C but when switched to 39°C the cells express a number of markers characteristic of mature hair cells [14]. In this study we have investigated the expression of several integrins in OC-2 cells and their role in controlling the differentiation processes of OC-2 cells. We demonstrate that among the integrins detected in OC-2 cells the expression of β3 is directly related to the production of myosin VIIa, a marker of differentiated hair cells.

The article "β3-integrin is required for differentiation in OC-2 cells derived from mammalian embryonic inner ear" was published in 2012. Journal: BMC Cell Biol.

## Results

### Increased integrin expression in differentiated OC-2 cells

To confirm that OC-2 cells grown at 39°C for 2 weeks had differentiated, myosin VI and myosin VIIa levels were examined by Western blot analysis. As has been shown previously [14], differentiated OC-2 cells increased their expression of both myosin VI and VIIa (Figure 1A) (*P *< 0.01) with respect to undifferentiated cells.

**Figure 1:** **Integrin expression profiles are altered after OC-2 cell differentiation**. **(A) **Western blot analysis of myosin VI and myosin VIIa levels in OC-2 cells grown at 33°C and 39°C. Both myosin VI and VIIa levels were increased significantly in cells grown at 39°C cells in comparison with those incubated at 33°C. Bar graphs represent densitometric results of mean relative values of myosin VI and myosin VIIa levels ± s.e.m. HSC-70 provided the loading control. **(B) **Undifferentiated (33°C) and differentiated (39°C) OC-2 cells were analysed by FACS for the integrin subunits α6, β1, αv and β3. Levels of β1-, αv- and β3-integrin subunits were increased significantly in differentiated OC-2 cells when compared with undifferentiated OC-2 cells. α6-integrin surface expressions levels did not change between the two cell phenotypes. Bar graph represents mean fluorescence units of the various integrin subunits ± s.e.m.; n = 3 independent experiments. White bars = cells at 33°C, black bars = cells at 39°C cells; nd = no significant difference, *P < 0.05, **P < 0.01.

FACS and Western blot analysis were utilized to quantify the relative changes of expression of the integrin subunits during the differentiation of OC-2 cells. OC-2 cells were screened for integrin expression and the integrin subunits α6, αv, β1 and β3 were detected (Figure 1B) but not α1-, α2-, α5- and β4-integrin subunits (data not shown). The expression of α6-integrin subunit was not significantly different between undifferentiated and differentiated OC-2 cells. In contrast, αv- and β1-integrin surface levels were increased in differentiated OC-2 cells when compared with undifferentiated OC-2 cells (*P *< 0.01) (Figure 1B). No expression of β3-integrin was observed in undifferentiated OC-2 cells but this receptor was expressed after the OC-2 cells had undergone differentiation (*P *< 0.01). Similar results were obtained when total protein levels of these integrin subunits were examined by Western blot analysis (data not shown). To verify our in vitro findings, RT-PCR for the integrin subunits α6, αv, β1, β3 and β4 (as a control) was performed on RNA isolated from cochlear tissue of adult mice (Figure 2). All integrin subunits examined were expressed in mouse cochlear tissue, to varying levels, apart from β4-integrin, which also was not expressed on OC-2 cells.

The article "β3-integrin is required for differentiation in OC-2 cells derived from mammalian embryonic inner ear" was published in 2012. Journal: BMC Cell Biol.

**Figure 2:** **Integrin expression profiles in the Organ of Corti**. RT-PCR of RNA isolated from organ of Corti of adult mice. Bands at the predicted molecular weight are visible for integrin β1, β3, αv, α6 and β-actin but not for integrin β4. cDNA was omitted for the negative control.

### Time course of integrin expression profiles during differentiation

Having shown that differentiated OC-2 cells had increased expression of αv, β1 and β3-integrin, we analysed the pattern of integrin expression over the 14 day differentiation period. OC-2 cells, cultured at 33°C, were transferred to 39°C and integrin expression was examined every 2 days for 14 days, when the cells had fully differentiated. Unsurprisingly, α6-integrin levels did not alter during the 14 day differentiation period (Figure 3A). αv-integrin expression levels remained similar to levels seen at 33°C cells for the first 4 days during differentiation. By day 6 of differentiation, αv-integrin expression levels increased to the levels observed in fully differentiated OC-2 cells (Figure 3B), and remained so until OC-2 cells were fully differentiated (day 14). However, we did observe that at day 10 of differentiation, the level of αv-integrin expression was increased to a level above that found in fully differentiated OC-2 cells.

**Figure 3:** **αv-integrin expression profiles change during differentiation**. Expression of **(A) **α6-integrin and **(B) **αv-integrin were examined by FACS at days 2, 6, 10 and 14 during the differentiation process. The differentiating cells ('dif' red line) were compared to undifferentiated ('33' green line) and fully differentiated cells ('39' red line). α6-integrin expression profiles did not change throughout the time course. αv-integrin expression profiles show an increase at day 6 and are at comparable levels with fully differentiated OC-2 cells at day 14 with an apparent even higher level at day 10.

β1-integrin expression increased from day 2 of differentiation when compared with undifferentiated OC-2 cells. β1-integrin levels gradually increased until day 10, at which time β1-integrin surface expression was comparable to levels observed in fully differentiated OC-2 cells (Figure 4A). It was noted that throughout the early stages of differentiation (day 2-8), a small population of differentiating OC-2 cells expressed β1-integrin at a level comparable with fully differentiated OC-2 cells. No surface expression of β3-integrin was seen during the first 2 days of the differentiation process, but by day 4, expression of this integrin increased with time, reaching the level of expression observed in differentiated OC-2 cells by day 12 (Figure 4B). Western blot analysis of all the described integrin subunits showed similar patterns of integrin expression during the differentiation process, while the increase in myosin VIIa and myosin VI that occurs with differentiation (Figure 1A) started being evident from day 8 and day 12 respectively (data not shown).

The article "β3-integrin is required for differentiation in OC-2 cells derived from mammalian embryonic inner ear" was published in 2012. Journal: BMC Cell Biol.

**Figure 4:** **β1 and β3-integrin expression profiles change during differentiation**. Surface expression of **(A) **β1-integrin and **(B) **β3-integrin was examined by FACS at days 2, 6, 10 and 14 of the differentiation process The differentiating cells ('dif' red line) were compared to undifferentiated ('33' green line) and fully differentiated cells ('39' red line). Increase of β1-integrin expression profile is visible from day 2 and it reaches the level of differentiated cells by day 10. β3-integrin expression which is undetectable above the Ig signal up to day 2, becomes visible at day 6 and gradually reaches the differentiated levels at day 14.

### Functional correlation between integrin expression and myosin VIIa levels

Having shown that changes in the integrin expression profiles during differentiation coincided with changes in myosin VI and myosin VIIa levels, we wished to confirm a functional role for these integrins in this process. Fully differentiated OC-2 cells were transfected with siRNA targeted specifically to either αv-, α6-, β1- or β3-integrin subunits or a scrambled control siRNA, followed by analysis of myosin VIIa levels. We optimised the time of maximum effect of siRNA on the respective protein surface expression (24 hrs) and confirmed siRNA treatment had no effect on cell proliferation and was non-toxic to the cells (data not shown).

Western blot analysis showed that siRNA inhibition of all integrin subunits significantly reduced the level of expression of myosin VIIa in comparison with fully differentiated OC-2 cells, to levels similar to those observed in undifferentiated OC-2 cells (*P *< 0.01). Myosin VIIa levels were decreased most effectively in the presence of αv and β3-integrin siRNA (Figure 5A). To investigate the specificity of action of the integrin subunits we have measured the effect of some of the integrin siRNA on the expression of other integrin subunits. All integrin siRNAs, but not scrambled siRNAs significantly reduced the surface expression of their respective proteins and in some cases also other integrins. For example (Figure 6) β3-siRNA caused a significant reduction of surface expression of β3, αv, β1 but not α6. Other examples of non-significant effect of siRNAs were α6-siRNAand αv-siRNA on β1 expression (data not shown). These data indicate that the effect of the siRNAs is specific but there is interdependency in the surface expression of different integrin subunits.

The article "β3-integrin is required for differentiation in OC-2 cells derived from mammalian embryonic inner ear" was published in 2012. Journal: BMC Cell Biol.

**Figure 5:** **β3-integrin is a marker for OC-2 cell differentiation**. **(A) **Western blot analysis of myosin VIIa expression in 39°C OC-2 cells untreated or after treatment with either scrambled (Scr), β1-, α6-, αv- and β3-integrin siRNA. Treatment with all siRNAs reduced myosin VIIa levels significantly when compared with untreated OC-2 cells or OC-2 cells treated with scrambled siRNA. **(B) **Undifferentiated OC-2 cells transduced with human β3-integrin (+hβ3) had similar levels of surface β3-integrin to differentiated (39) OC-2 cells. Furthermore, analysis of the expression of myosin VIIa showed it was increased significantly in OC-2 cells transduced with human β3-integrin (+hβ3) cells compared with undifferentiated (33) cells. Bar graphs represent densitometric results of mean relative values of myosin VIIa levels ± s.e.m. HSC-70 was used as a loading control. *P < 0.05, **P < 0.01. n = 3 individual experiments.

**Figure 6:** **Effect of β3-integrin-siRNA treatment on integrin surface expression**. Differentiated OC2 cells were treated with β3-siRNA and assayed by FACS for expression of surface integrins. The data is compared to integrin expression levels in normal differentiated cells (39°), differentiated cells exposed to scrambled siRNA sequences (siRNAβ3) and undifferentiated cells (33°). Exposure to β3-integrin-siRNA resulted in a significant reduction of the surface expression of β3, β1- and αv- to levels similar to those of undifferentiated cells. There was no significant effect of scrambled siRNA sequences on any integrin expression and β3-integrin-siRNA did not significantly affect α6-integrin providing further evidence for the specificity of the siRNA inhibition.

Having shown that β3-integrin diplayed the most dramatic change in integrin expression during madifferentiation of the OC2 cells and that knockdown of this integrin was the most effective at reducing the expression of myosin VIIa, we over expressed β3-integrin in undifferentiated OC-2 cells to generate a phenotype similar to fully differentiated OC-2 cells. Retroviral transduction of undifferentiated OC-2 cells with human β3-integrin was confirmed by FACS analysis (Figure 5B) and showed surface expression levels similar to those observed in fully differentiated OC-2 cells. This over expression of β3-integrin, in turn, increased the expression of myosin VIIa to levels similar to those in fully differentiated OC-2 cells. Indeed, myosin VIIa levels were increased significantly in transduced cells when compared with undifferentiated OC-2 cells. The effect of over expression of human β3-integrin on other integrin expression patterns was examined by FACS analysis. α6-integrin surface levels did not change in response to increased β3-integrin, whereas αv-integrin, and, to a lesser extent, β1-integrin showed increased surface expression after transduction with human β3-integrin (data not shown).

The article "β3-integrin is required for differentiation in OC-2 cells derived from mammalian embryonic inner ear" was published in 2012. Journal: BMC Cell Biol.

## Discussion

In this study we have utilised the OC-2 cell line to study the role of integrin proteins in the regulation of differentiation of this cell line. The OC-2 cells display only some of the characteristics of the cells of the organ of Corti from where they have been derived. However, they do have a temporal pattern of gene expression that reflects the developmental processes observed in the organ of Corti. Therefore we believe the findings reported here can be considered of significance for the understanding of the maturation and/or regeneration processes of the organ of Corti. In this study we have observed in differentiating OC2 cells a differential pattern of developmental expression of integrin subunits ranging from no change as in α6, to an increase from sub-detectable levels to higher levels for β3. Other variations included a peak of αv expression at day 10 above the level of the fully differentiated cells and the presence of a sub-population of differentiating cells with high β1 expression. Taken as a whole these expression patterns indicate a complex relationship between integrin expression and the differentiation of OC2 cells. In this study we have began to unravel this complexity by establishing a temporal and functional relationship between the expression of integrins and the expression of the mature hair cell markers (summarised in Figure 7).

**Figure 7:** **Graph of changes in expression levels of integrin subunits and myosin VIIa during OC-2 cell differentiation**. Schematic time course graph showing fluorescence values of αv-, α6-, β1- and β3- integrin subunit surface expression measured by FACS and chemiluminescence values of the hair cell marker myosin VIIa in OC-2 cells measured by Western blot, over the 14 day differentiation process.

The article "β3-integrin is required for differentiation in OC-2 cells derived from mammalian embryonic inner ear" was published in 2012. Journal: BMC Cell Biol.

This study did not aim to identify all the possible integrins that are expressed by OC-2 and it is plausible that other integrins may also be expressed and affect differentiation of OC-2 cells. Our interest was directed at verifying our hypothesis that the expression of some integrins can be functionally correlated to the expression of hair cell differentiation markers. Our data demonstrate at least one integrin subunit (β3) plays such role in the expression of the hair cell differentiation marker myosin VIIa. Expression of β3 integrin appears to be both necessary, as demonstrated by the decrease of expression of myosin VIIa in differentiated OC-2 cells exposed to β3-siRNA, and sufficient as indicated by the expression of myosin VIIa in undifferentiated cells virally transfected with β3-integrin gene. Our siRNA data and β3-transfections data also indicate that the expression of one integrin subunit can affect the surface expression of other integrins subunits. The specificity of this latter effect is substantiated by the fact that scrambled siRNA did not affect the expression of any integrin subunits and some integrin siRNA (e.g. β3) did not inhibit the expression of specific integrins (e.g. α6, Figure 6). A full investigation of all the respective inhibitory effects of integrin siRNA on other integrin subunits was not within the scope of this study. However, of our data does suggest that this would be a worthwhile aim. The transcriptional expression of one integrin subunit could affect the surface expression of another integrin by a number of mechanisms ranging from transcriptional regulation of gene expression to post-translation modulation of integrin receptor assembly. The β3 subunit predominantly dimerises with αv to form a functional integrin receptor [8]; further studies would be required to establish whether the β3 subunit competes with other beta subunits to dimerise with αv, or whether the observed increase in αv is sufficient to form additional functional dimers with β3.

Interaction between integrins and cytoskeletal proteins, including myosins, has been reported in several systems including the inner ear[15]. What is of particular interest with respect to the organ of Corti is that the differentiation of the precursors of hair cells and supporting cells involves detachment from the basilar membrane which is composed of extracellular matrix proteins recognised by integrin complexes [5,16]. The data described in this paper, if confirmed in the organ of Corti, would help to elucidate a central mechanism of the developmental processes of the inner ear and may lead to a better understanding of the lack of regeneration of inner ear tissue following injury. The OC-2 cells represent a good model for testing some of the potential mechanism of integrin involvement in hair cells development. However to more faithfully mimic the events that occur in vivo it would also be necessary to reproduce the changes in extracellular proteins that have been shown to occur in the organ of Corti during development[17]. While our data demonstrate a clear link between integrin expression and OC-2 cell differentiation, it would be premature to utilise our data to speculate on the exact mechanisms of the development of hair cells. To better understand the differentiation mechanisms that take place in the OC-2 cells, further work will be conducted to elucidate the relationship between integrin subunit expression and other hair cell markers such as the alpha 9 subunit of the acetylcholine receptor [18] as well as other signalling proteins known to be associated with integrins [9]. Ultimately, it will be necessary to demonstrate that the developmental mechanisms observed in OC2 cells also take place in the organ of Corti.

The article "β3-integrin is required for differentiation in OC-2 cells derived from mammalian embryonic inner ear" was published in 2012. Journal: BMC Cell Biol.

## Conclusions

We have demonstrated that in OC-2 cells there is causal relationship between β3- integrin expression and the expression of the hair cell differentiation marker myosin VIIa. These data could reflect similar events occurring during the development of the organ of Corti.

## Methods

### Antibodies

Antibodies against α1, α2, α5 and β1-integrin subunits for flow cytometric analysis were a kind gift from B. Chan (Universtiy of Western Ontario, Canada). Biotinylated β3-integrin antibody was purchased from Pharmingen (Bedford, UK). αv-integrin antibody was purchased from Chemicon International (Harrow, UK). α6-integrin antibody was purchased from ABD Serotec (MorphoSys Ltd, Kidlington, UK). β4-integrin antibody was purchased from AbCam (Cambridge, UK). HRP and FITC-conjugated anti-rabbit, anti-rat and anti-mouse antibodies were all purchased from Jackson Immuno Research Labs (Baltimore Pike, PA, USA) or from Biosource (Nivelles, Belgium). Myosin VI and myosin VIIa were purchased from Abcam (Cambridge, UK). For Western blot analysis, αv and β1-integrin antibodies were purchased from Chemicon International. β3-integrin and HSC-70 antibodies were obtained from Santa Cruz (Wiltshire, UK).

### OC-2 cell culture

OC-2 cells (gift from Prof M. Holley, Sheffield University, UK) [18] were cultured at 33°C in a 5% CO_2 _atmosphere in DMEM + 10% FCS + 10% glutamine in order to express the immortalisation gene, small tumour antigen (Tag). Under these conditions the cells can be passaged multiple times by detaching the cells from the flasks with trypsin/EDTA (1x T3924 Sigma). To induce differentiation, the cells were cultured at 39°C in 5% CO_2 _in DMEM + 10% FCS + 50 U/mL^-1 ^IFNγ + 10% glutamine for 14 days to inactivate the immortalisation gene. The phenotype of undifferentiated and differentiated OC-2 cells was confirmed by examining the cellular morphology and expression of myosin VI and myosin VIIa expression levels, prior to use in experiments.

The article "β3-integrin is required for differentiation in OC-2 cells derived from mammalian embryonic inner ear" was published in 2012. Journal: BMC Cell Biol.

### Flow cytometry analysis

Single cell suspensions of undifferentiated and differentiated OC-2 cells were incubated with either anti-α1, -α2, -α5, -α6, -αv, -β1, -β3 or -β4 antibodies followed by incubation with a FITC-conjugated secondary antibody. Cells were then washed and resuspended in FACS buffer (0.1% BSA in PBS) and analysed for fluorescence using a Becton Dickinson FACS Calibur flow cytometer. For negative controls, IgG matched isotype controls were used. Flow cytometry experiments were repeated 3-9 times.

For retroviral transduction experiments, transduced cells were screened by FACS analysis using a human β3-integrin antibody, LM609 (BD Pharmingen), to determine the level and efficiency of transduction.

### OC-2 retroviral infection

Undifferentiated OC-2 cells were grown to 60% confluency and transduced with retrovirus expressing either the human β3-integrin (gift from J. Marshall, QMUL, London) or an empty expression cassette, for 48 h at 33°C. After 48 h incubation, the viral medium was removed and replaced with OC-2 cell culture medium followed by further incubation for 48 h. OC-2 cells infected with β3-integrin were selected from the non-infected cells by magnetic bead sorting (Dynal, Invitrogen, UK) using the antibody against β3-integrin (LM609). Cells were either lysed for Western blot analysis of myosin VI and myosin VIIa or trypsinised for FACS analysis of mouse and human β3-integrin surface levels.

### Western blot analysis

Undifferentiated and differentiated OC-2 cells were grown to 70-80% confluency and lysed using RIPA buffer. Equal amounts of protein from each cell type were analysed by SDS-PAGE followed by transfer to nitrocellulose membranes (Hybond-ECL, Amersham Biosciences, Buckinghamshire, UK). Membranes were blocked for 1 h in either 5% milk-PBS-Tween (0.05%) followed by incubation with antibodies against αv-, α6-, β1- and β3-integrin or myosin VI and myosin VIIa, overnight at 4°C. Membranes were washed 3 times with PBS-Tween (0.05%) followed by incubation with an HRP-conjugated secondary antibody for 1 h at room temperature. Chemiluminescence was detected by exposure to high performance chemiluminescence film (Amersham Biosciences, UK). Densitometric readings were obtained using Lab Images software. HSC-70 was used for a loading control.

The article "β3-integrin is required for differentiation in OC-2 cells derived from mammalian embryonic inner ear" was published in 2012. Journal: BMC Cell Biol.

### RT-PCR

Adult mice (Mus-musculus CBA/Ca) were killed by cervical dislocation according to Home Office regulations. Total RNA was isolated both from mouse cochlear tissue and from differentiated and undifferentiated OC-2 cells using the RNeasy mini kit from QIAGEN (Bio-Rad, Hercules, CA, USA). RNA was reverse transcribed using the Superscript III First-strand Synthesis kit (Invitrogen). The primers used to identify the different integrins were as follows (F = Forward, R = Reverse): α6 F: AGGAGTCGCGGGATATCTTT; α6 R 5'- GTAACAAAGCTCAGGGCTGC; αv F: CCAGCCCATTGAGTTTGATT αv:R: AAATCTTCAATGCCGTCACC; β1 F: GCTCCTCTTCCCCTCCATAC; β1 R GTAACAAAGCTCAGGGCTGC; β3 F GCTACAAACACGTGCTGACG; β3: R GAGGCAGAGTAGTGGTTGTCG β4 F GATGCCTACCCAGTCCTCAA β4 R TTCATAGGGCCACTCCAGAC.

The reaction conditions of the above sequences were as follow: denaturation at 94°C for 2 min; extension at 58°C for 45 s; and annealing at 72°C for 60 s for thirty cycles. PCR products were separated on a 1% agarose gel by electrophoresis for 1 h at 100 V.

#### Integrin siRNA transfection

One day prior to transfection, differentiated OC-2 cells (39°C) were counted and seeded at 1 × 10^5 ^cells per T-25 flask in medium without antibiotics to generate a 50-60% confluent monolayer on the day of transfection. A pool of four different oligonucleotides (siRNA SmartPool, Dharmacon, USA) was used to knockdown each single integrin mRNA efficiently. The integrin oligonucleotide sequences were as follows (5'-3'):**α6**: UUAACCUUGAGGCAUAUCCUU; UUGUUCUACACGGACGAUCUU; UUAAUGUAGACGUAAACUGUU; UGAUCCACCAAGCUACUCCUU. **αv**: UACUCAACGGUCUUUGUGCUU; AAAUGCUAGGGUACACUUCUU; UUCACGUACAGGAUUGCGCUU;UCGAUUGGCAGGUUCUUGUUU. **β1**: UCAUUCAUCAAAUCCGUUCUU; UUAAUGUAAACUUCUGUGGUU; UGAAACUUGGGAUCUGUGCU; GUAAUCUUCAGCCCUCUUGUU. **β3**: UAUACAGCGGGUUGUUUGCUU; UUCUCCUUCAGGUUACAUCUU; GUAGUAGCCAGUCCAGUCCUU; UAGUUUCUCAGUCAUCAGCUU

For one T-25 flask of cells, 2.5 μl of a 40 μM stock oligonucleotide solution was mixed, in a tube, with 182.5 μl of OPTIMEM to give a final volume of 185 μl. Oligofectamine, 3 μl (Invitrogen, Paisley, UK) was diluted in OPTIMEM to give a final volume of 15 μl and incubated for 5-10 min at room temperature (RT). The two solutions were then combined together to give a final volume of 200 μl and allowed to form a complex by incubating for 15-20 min at RT. The solution was added to each T-25 flask containing the cells to be transfected in 800 ul serum free medium. Cells were returned to the incubator set at 37°C in 8% CO_2_. Four hours after transfection, 500 μl of cell culture medium containing 3X the normal concentration of serum without antibiotics was added to each flask. Gene knockdown was assessed by FACS analysis 24 h after transfection. After verification of positive knockdown by FACS analysis, protein and RNA extraction was performed. Transfection with a scrambled oligonucleotide was carried out as control and shown to have no change on integrin expression

The article "β3-integrin is required for differentiation in OC-2 cells derived from mammalian embryonic inner ear" was published in 2012. Journal: BMC Cell Biol.

#### Statistical analysis

Statistical significance was calculated using Student's t-test. *P *< 0.05 was considered statistically significant.

## Competing interests

The authors declare that they have no competing interests.

## Authors' contributions

IB carried out all the experiments, designed or contributed to the design of the experiments and to the preparation of the manuscript. SOC contributed to the preparation of the manuscript and to the initial analysis of integrin expression in the inner ear. IRH contributed to the design of the experiments and the preparation of the manuscript. AF contributed to the design of the experiments and the preparation of the manuscript. LER designed and supervised the majority of the experiments and contributed to the preparation of the manuscript. All authors read and approved the final manuscript.
